# Shape Prediction of Nasal Bones by Digital 2D-Photogrammetry of the Nose Based on Convolution and Back-Propagation Neural Network

**DOI:** 10.1155/2022/5938493

**Published:** 2022-01-11

**Authors:** Ho Nguyen Anh Tuan, Nguyen Dao Xuan Hai, Nguyen Truong Thinh

**Affiliations:** ^1^Human Anatomy Department, Pham Ngoc Thach University of Medicine, Vietnam; ^2^Department of Mechatronics, Ho Chi Minh City University of Technology and Education, Vietnam

## Abstract

In rhinoplasty, it is necessary to consider the correlation between the anthropometric indicators of the nasal bone, so that it prevents surgical complications and enhances the patient's satisfaction. The penetrating form of high-energy electromagnetic radiation is highly impacted on human health, which has often raised concerns of alternative method for facial analysis. The critical stage to assess nasal morphology is the nasal analysis on its anthropology that is highly reliant on the understanding of the structural features of the nasal radix. For example, the shape and size of nasal bone features, skin thickness, and also body factors aggregated from different facial anthropology values. In medical diagnosis, however, the morphology of the nasal bone is determined manually and significantly relies on the clinician's expertise. Furthermore, the evaluation anthropological keypoint of the nasal bone is nonrepeatable and laborious, also finding widely differ and intralaboratory variability in the results because of facial soft tissue and equipment defects. In order to overcome these problems, we propose specialized convolutional neural network (CNN) architecture to accurately predict nasal measurement based on digital 2D photogrammetry. To boost performance and efficacy, it is deliberately constructed with many layers and different filter sizes, with less filters and optimizing parameters. Through its result, the back-propagation neural network (BPNN) indicated the correlation between differences in human body factors mentioned are height, weight known as body mass index (BMI), age, gender, and the nasal bone dimension of the participant. With full of parameters could the nasal morphology be diagnostic continuously. The model's performance is evaluated on various newest architecture models such as DenseNet, ConvNet, Inception, VGG, and MobileNet. Experiments were directly conducted on different facials. The results show the proposed architecture worked well in terms of nasal properties achieved which utilize four statistical criteria named mean average precision (mAP), mean absolute error (MAE), *R*-square (*R*^2^), and *T*-test analyzed. Data has also shown that the nasal shape of Southeast Asians, especially Vietnamese, could be divided into different types in two perspective views. From cadavers for bony datasets, nasal bones can be classified into 2 morphological types in the lateral view which “V” shape was presented by 78.8% and the remains were “S” shape evaluated based on Lazovic (2015). With 2 angular dimension averages are 136.41 ± 7.99 and 104.25 ± 5.95 represented by the nasofrontal angle (g-n-prn) and the nasomental angle (n-prn-sn), respectively. For frontal view, classified by Hwang, Tae-Sun, et al. (2005), nasal morphology of Vietnamese participants could be divided into three types: type A was present in 57.6% and type B was present in 30.3% of the noses. In particular, types C, D, and E were not a common form of Vietnamese which includes the remaining number of participants. In conclusion, the proposed model performed the potential hybrid of CNN and BPNN with its application to give expected accuracy in terms of keypoint localization and nasal morphology regression. Nasal analysis can replace MRI imaging diagnostics that are reflected by the risk to human body.

## 1. Introduction

In today's society, appearance plays a crucial role and affects almost all, as a reaction to the need for beauty and to ensure the symmetry of the face, especially the nose, which is the protruding component of the human face that has gained the interest of widespread science in the process of recognizing individuals. Rhinoplasty is supposedly known as the alternation, restoration, or reconstruction of the nose. Reconstructive surgery changes the appearance of the nose for beauty purposes and restores the form and functions of the nose. One of the primary reasons that people require rhinoplasty not only for beauty but also the nasal bone is the thinnest and softest of the facial bone [1], in which 23.2% of the facial fracture from a retrospective review made of 151 patients over a 4-year period was nasal bones, shown by Alvi et al. 2003 [2]. Furthermore, forty-nine percent of broken facial nasal bones were immediately affected when drivers or passengers were involved in a collision, analyzed by Cormier and Duma 2009 [3]. From Byun et al., male patients surpassed the number of female patients by 3.3 times for the age of 20. The most common cause of injury overall was abuse [4]. Nasal injuries can be mentioned as penetrating trauma-affected by bombs, war, or breathing problems, could be a deviated nasal septum or a sinus, or even treats birth defects problem like cleft palate disease [5] especially cancer patients with necrotic wounds that need surgery [6, 7]. The other factor is genetic inheritance of the dorsal humps or acquired during growth [8]. For almost all people, these naturally occurring bumps on the nose have nothing unhealthy or risk [9], while some feel not confident with dorsal humps appearing. Moreover, according to the concept of the Eastern, especially Asian, morphology of nose surgery depends on the desire and purpose to change fortune [10]. As a result, in addition to correcting a visible facial defect caused by the nose, the nasal bone is critical in balancing the proportion of the face between the need for adaptation and the nose and embellishing for self-confidence. However, its diverse shape and human presence are correlated with life phases, gender, race [11–15], and body mass index (BMI) [12]. The nose shape is designed to regulate its efficiency as a sense of smell as well as to play an important role in breathing.

In the cutting-edge of the technological revolution, diagnostic is taken easily and flourished in rhinoplasty. With modern clinical techniques of development, many studies have helped people to diagnose the bone structure through the epidermis without needing to do surgery. Thanks to digital medical images, the statistical analysis combines vision machine with computer aid, plastic surgery now can be performed much easier. The doctor not only detail described anatomical variation of nasal septum by digital scanned of cadaver specimens [16] but also analysis the development of nasal septum according to specific age and gender by magnetic resonance imaging (MRI) [17]. Beyond that, computerized tomography (CT) scan was used efficiently to measure and estimate nasal septal cartilage area [18]. CT scans have been an advantage for medical treatment and diagnostics. However, following the nearest researches, ionizing radiations impose risks to human health including occupational risk, patient safety, and also the environment [19]. Therefore, CT scans are also harming patients with ionizing radiation which is a known human carcinogen [20], resulting in a possible public health disadvantage, with anatomical visualization intended to implement diagnostics, improve outcomes, and prevent invasive surgery. Growing health issues around radiation hazards are now driving forward efforts to limit preventable CT scans and possibly reduce radiation exposures [21]. Therefore, facial anthropometric analysis is one of the most commonly used alternative method for lowering operating costs while improving patient welfare [22]. This study presents an efficient method to analyze facial anthropometric with the support of deep learning in the diagnosis of nasal morphology with dependence various. As a result, this study hopefully contributes a rapid and precious model applying in surgical preparation and nose modeling. Based on the result, defects under surface skin layers had been located by the surgeon that can limit the minimum damage and do not leave the scar after surgery. Facial anthropometric analysis [23] with computer aid is almost applied in many fields might be mentioned as diagnosing medical images, surgical planning [24], facial reconstruction surgeries, facial security [25], and also forensic investigation [26]. CNNs used an indirect anthropometry technique on approach research to provide the best digital image diagnoses where conventional calculation is restricted due to the need to measure on human skin using a purely manual measuring instrument, and since human skin is a soft surface, the ruler sinks into the skin, leading error to be recorded. On the other hand, it would not necessitate overt interference by medical personnel or have an effect on the human. Modeling is an important tool for understanding the linkages between nasal bone structure and as well as for predicting nasal morphology under a self-consistent framework. Machine learning models, such as the most widely used the artificial neural networks, have been used to efficiently classify as a feature of its influencing factors for rapidly depicting the interdependence between the nasal bone and facial landmark, thereby have been considered a better choice for nasal bone detection. For instance, fracture prediction by CNN [27] and R-CNN [28] is considered critical to early warning and well treatment of planning surgery. Indirect measurement models with CNN have received extensive attention over the last decades; Anjit and Rishidas [29] show the facial recognition model composing with two-layer deep CNN for feature extraction and SRC for classification. A variety of machine learning techniques have been used to predict nasal problems, such as the back-propagation neural network (BPNN) for the identification of the nasal bone [30], the long short-term memory neural network (LSTM) in SAHS event detection based on breathing [31], the random forest (RF) [32], and the support vector machine (SVM) [33]. Hybridization approaches integrating different machine learning techniques [34] have also been explored in recent years to improve nasal bone morphological prediction reliability and accuracy, with satisfactory morphology results. In this study, the hybrid of CNN and BPNN proposed is an interesting model enabled to not only locate multiple keypoint attributes at once by also investigating the association between anthropometry and morphometric of the nasal bones by determining major facial landmarks and the other additional body indexes. The positions of landmarks and some specific distances measured on cadavers were correlated with the location of nasal landmarks on the facial surface. The predicted result can be visualized in a 2D map.

Following anthropometric, facial landmarks (keypoints) are used to localize and represent salient regions of the faces which can be easily determined by Euclidean geometry on the projection plane. In addition, indicated by Farkas et al. [35] that classical landmarks obtained by direct anthropometry would typically also be obtained by 2D-photogrammetry. Moreover, the dominant technique for defining the various anatomical features was the use of direct anthropometric, while actually, the most generally employed method is indirect anthropometry, 2D-photogrammetry instead of direct anthropometry pointed out by Farkas et al. [36–38]. Their method described a widely used series of measurements to describe the human face. The anthropometric analysis is essential to provide a detailed description of face anthropometry and its various important applications to define nasal morphology in terms of projective measurements, tangential measurements, and angular measurements. Nasal bone morphology and its correlation with the other body indexes is a central part of the anthropometric analysis. The bony shape could be classified by different types in distinct ways. For instance, in the profile view, Hwang et al. [39] proposed the original shape of the nasal bone, while Uzun and Fikri [40] are classified the original into the easier way. On the other hand, Lazovic et al. showed the nostril models and nasal profiles in young Turkish by sex [41], meanwhile Sugawara [42] described properly organize their procedures inside the radix and bone and cartilaginous vaults which classify the nasal shape into two morphologies which are “V shape” and “S shape” from measured distances on Caucasian bony. In this study, analysis of Vietnamese nasal bone shape had been presented and classified following two perspective looks as Hwang et al. (2005) and followed by Lazovic (2015). However, we force open surgery to prolong the patient's recovery process and it is difficult to collect data due to muscle components and soft tissue cover surrounding the nasal bones, so it needs to be analyzed from the nose's surface. On the other hand, in the fields of otolaryngology and anthropology, as there are distinct variations between races in form and scale of the nose, there are undoubtedly certain differences in the nasal bone's shape and sizes. The shape of the various Turkish's nose is a sign indicating specific race, age, and sexual dimorphism which introduced by Lazovic et al. [41], and it is possible to pass through the parameters of the human index; these characteristic features to diagnose the morphology and also the type of nose that one possesses. Hence, it is possible to predict the size and morphology of the nasal bones through physical indicators of the body. Secondly, based on Sugawara's research on nasal morphology in typical rhinoplasty of Asian [42] by topological analysis method to show the correlation of nose shape based on the shape of the external surface of the nose, the method of collection image acquisition, simulation by manual photo editing software by physician experience, shows the change of nose before and after surgery from straight and horizontal images and also shows the correlation of fat layer, muscles, and nasal bones through the experiments. However, it should be noted that detecting nasal anthropology by hand was laborious, time-consuming, and nonrepeatable in the preceding experiments. Advances in neural networks continue to separate nasal skeletal into distinct groups using linear measurement and angular dimensions. As a result of analyzing the previous related works, the importance of using hybrid deep learning in regression nasal bone morphology based on human body variables may be studied in order to improve and accelerate the diagnostic process for determining nose shape rather than utilizing handle photo may be studied. Furthermore, good manipulation of these contributing parameters can simulate and improve the morphology of the effect on a 2D snapshot. Furthermore, based on participant data, this research concentrates on remarks about the typical nasal bone form of the Asian group based on external 2D shapes provided significantly. The generated nasal sizes are automatically based on a photograph without fixing the head, which is a sophisticated system with the trained model. Following Introduction, this study is organized to outline the material and methods in Section 2 and introduce the methods and feature definition of nasal anthropology in Section 3.  Section 4 presents the hybrid of CNN and BPNN. Experiments and results are shown and remarked in Section 5.

## 2. Materials and Methods

### 2.1. Data Collection

The study is aimed at using digital images to be able to generate the facial landmark based on nasal anthropology most accurately and predict its morphology. The procedure and computer simulation process are important to choose suitable photographs that may compare the exact model provided by the parameters derived by different human indexes. Practically, firstly, patients on project have been conducted to determine facial landmarks with caliper and using stainless steel ruler for reference; however, these custom works, though, are often time-consuming and costly. Therefore, the hybrid of CNNs and BPNN-aided diagnostic for nasal anthropology from digital 2D images is required; facial landmarks on human's skin could be detected in a second with high precise instead of traditional methods. However, the range by which a picture is taken influences the face's position in the shot. Image distortion will appear when the focal length of the lens is less than 50 mm. Moreover, for intraoperative photos, a macrolens is especially useful and recommended when the focal length of the lens is greater than 70 mm [42]. The camera Canon ILCE-7M2 was used in this study. The image for image processing was captured by custom setting at 1/60 second, and aperture inlet is f/6.3. Focal length of the lens is 55 mm, ISO 200. The required participant must never have facial plastic surgery and are not affected by eye problems in which they asked to sit still in a position to avoid muscle fatigue, or position moving while cameras obtain pictures in the short period time. This work helps hold statement of the participant at the same moment and reduce as much as possible image round error. Cameras are placed in the same mechanical system which the first camera is shot straight and perpendicular projection with frontal plane. The focus point captured directly at the closest point from the camera lens is the nose tip (prm). The second camera is placed at the lateral plane, perpendicular to the median plane and the Frankfort horizontal plane indicated on the lateral face parallel to the ground. The focal length of the lens is the same distance as the human nose as the first camera. The third camera was placed on the basilar plane; it would adjust to catch the nostril at the bottom view. Efforts to capture images from objects were made to ensure true profile views in 3 frame-based settings. Participants were asked to keep their head in horizontal plane, coronal plane, and sagittal plane at the same time. However, photographer care is needed to avoid shaking. Therefore, the experiment was established with unification of the best shooting angle with constant focal length and shooting angle. These experiments make sure to not change their posture and keep their face in neutral emotion in the short period to ensure a true record of object measurement.

### 2.2. Datasets, Preprocessing, and Augmentation

In this research, experiments are set up and collected at the University of Medicine Pham Ngoc Thach by participants individually. The databases contain facial images by multiviews of partners with information of gender, ages, and Asia origin, specifically Southeast Asia. Data consisted of 3 different data files described in Table 1: Firstly, the entire study group (*N* = 2000) served with facial images by 3 perspective views in which front view, lateral view, and basilar view; the ratio of men and women, respectively, is 4.36% and 95.64%, with the age means 35.09 ± 11.56 year old as the training file in CNN for landmark detect. The procedure has one main configuration parameter, which is the size of the train and test sets. Image data of 2000 participants and augmented data have been separated into a training set with the size of 80 percent of means that the remaining 20 percent are allocated to the test set; this subject file has been used for landmarks defined by CNN training. Secondly, in total, data for 182 healthy participants were randomly analyzed. Image of 81 males (in which 44.5%) at the age 22.01 ± 1.39 and 101 females (in which 55.5%) with the age means 21.88 ± 1.68 was considered as the evaluate file. The mean BMI was 22.34 ± 12.8 with the minimum and maximum BMI were 18.2 kg/m^2^ and 32.7 kg/m^2^.

Finally, facial of 33 cadavers, 18 males (in which 54.5%) and 15 females (in which 45.5%), with an average age at 64.9 ± 13.9, have been collected as the same view of healthy humans both originally, and yet operation, combined with the body's input parameters was used to predict the nasal shape based on BNN. All input volumes were resized to 224 × 224 pixels with normalization of the pixel on volumes. Image processing had used to resize the height and width of the image at the same ratio. In addition, aggressive data augmentation is used to improve or enrich the variety of data [43], especially the data is lacking because of limited by the number of volunteers or participants and also prevent overfitting when evaluating model with reality. The method was used with the batch generator framework such as spatial augmentations, colour augmentation, noise or cropping that serve as input data for the processing, and measuring system shown as the framework of proposals in Figure 1. Finally, images have been normalized following this function:

(1) $$\begin{array}{c} {\text{opv}}_{h,w}=\frac{\left({\text{ipv}}_{h,w}/255\right)-0.5}{\sigma }, \end{array}$$

where opv_*h*,*w*_, ipv_*h*,*w*_, and *σ* are the output pixel value, input pixel value, and standard deviation, respectively.

### 2.3. Training Architecture: Nasal Shape Regression Based on Facial Anthropology

First of all, each picture will be taken with a stainless steel ruler with a scale of at least 1 mm with an error of 0.02 mm. Secondly, from figures, marked points were provided by the doctor and expert's medical evaluation. The evaluated figures will be numbered and labeled with markers as the testing data. The proposed system shown in Figure 2 is divided into 4 stages. In stage 1, the CNN model is used at first trained with characteristic features of the human nose in a semisupervised method with 2000 samples. Clinical specialists have hand-labeled facial landmarks marked for first training of CNN. The dataset would be collected including feature extruded and localization of feature map. Through CNN, the model allows the unlabeled dataset to be able to identify specific facial points by three related direction views of the photographs. After that, predicted values have been implemented on both 182 living humans; each error was used to update the set of values for the weight of layers until loss score accordingly decreases. The CNN stage is allowed to provide the relatively accurate position of testing objects, specifically the location of landmark points which expressed by (*X*, *Y*) and (*Y*, *Z*) coordinates. Qualified samples are returned to test the unlabeled dataset, evaluating the first point (*X*_1_, *Y*_1_) to *n*-point (*X*_*k*_, *Y*_*k*_) values from true labels associated with predicted labels of CNN. The trained model will be implemented to produce data about distance and face corners of specific enrollment points. Anthropological training for facial landmark detection carefully considerably chose 29 keypoints. With the same idea, cadavers were being measured including three perspective photos of pre- and postoperation; this work helps compare the relative of the nasal bone and the other factors such as skin thickness or subcutaneous fat. Stage 3 described the measurement from keypoints detected by CNN. Each landmark position on the face will be represented by a characteristic feature to help identify and build up the nose size with standard distance, which is shown in step 2 and step 3. The computer reconstructs the nose by mesh visualization based on the general size and shape of the nose, which is then compared to the actual size of the person. The neural network used the nose size as the input variable that predicts nasal bones from the physical body index, corresponding to the participant. In the final stage, thus, the model reach the appropriate accuracy level continues as a part of input layer combining with diverse variables listed as ages, genders [11, 13, 15], human body indexes (BMI) [44, 45], and race [46, 47] known as height and weight, estimating the relationship between the other factors with the shape of the nasal bone [48, 49]. As the result, based on CNN results on detection of the landmark, BPNN would diagnose the nasal bone shape properties with all facial features and body parameters.

## 3. Nasal Anthropology and Feature Extraction

According to human anatomy, the nasal bones have been enclosed and preserved by skin, ligament, and subcutaneous fat; the thickness of which may be substantially determined by CT or ultrasound. These approaches have now shown adverse impacts on public wellbeing. Photogrammetry is thus a standard and safety tool used to quantify features taken from photography, namely, the anthropometry method. Anthropometry is the bioscience of human body calculation [50]. Anthropometric results reveal several factors that focus on knowledge of the distribution of measures across population groups. In this study, shape of the nose is being recognized the anthropometric knowledge and using an artificial neural network to integral in the training model which expected result identify and distinguish various face easier. However, the nasal bone was hard to determine exactly the dimension of bone due to the thickness of the soft tissue known as the skin layer and subcutaneous fat because an individual is quantitative. Therefore, landmark points are the result of anthropometric evaluation with the identification of particular locations personally, described in terms of noticeable or tangible characteristics of the subject. For the ease for the patient and specialist, a visual history of the rhinoplasty procedure is provided with a comparable standard of excellence, beginning with the preoperative consultation and progressing after surgery. Although the anatomical structure of the nose consists of two main parts: the nasal bone and the nasal cartilage. Nasal bone shape based on the facial feature was the most interesting. Linear and angular measurements had been sequentially implemented on different perspective standard images based on the facial keypoint. Plastic and oral/maxillofacial surgery had been accepted as a method of determining the position and size of the nasal bones thanks to the palpable characteristics marked on the patient's skin surface known as keypoints or landmark points. Facial keypoints are interest features same as the others appearing on every human face. Face authentication, face recording in photographs and videos, face recognition, facial signals for medical care, and facial attribute inference are all helpful features in face analysis [51]. Indirect measurement on digital 2D-photogrammetry instead of using a calliper, compass, and casual equipment as direct measurement is much easier, faster, and given higher precision.

### 3.1. Metric Linear Measurement and Angular Measurements on Facial Surface

A reference plane called the Frankfort horizontal plane is used to measure the datum and minimize measurement errors. Frankfort horizontal plane is relatively parallel to the ground which is defined as a plane from the Porion (Po) to the Orbitale (Or) which is shown in Figure 1(b). This rule assures consistent pretreatment and posttreatment head position. Facial anthropometric points are symmetrical across the median plane in an uncertain size and uneven, a sequence of comparisons between any of these landmarks shall be carried out using carefully defined techniques and measurement equipment. In this study, the system uses a total of 29 landmark points including 10 pairs of these points that describe the pose of the nose. The landmarks with linear measurement and angular measurement are typically identified by abbreviations of corresponding anatomical terms which are described briefly in Figure 1. These locations of landmark have been collected and projected from 3 orthographic planes which 90 degrees perpendicular to each other. Anterior view as Figure 1(a), lateral view shown in Figure 1(b), and basilar view shown in Figure 1(c), along with line drawings, head position has the sign focus on lens focal length. As a result, measurements are repeated by the same individual are accurate and quantities of different individuals can be compared effectively. Points of reference reflect specific features on the face of each human and thus serve as the basis for the form of the correlation of facial parts; each person would have his/her characteristics on nose shape. Collected 2-dimension images are used to measure; however, the landmark points will not be on the same Cartesian coordinate system, leading to the need for a method to measure the distance 2 specific points in different planes.

The distance transform is a useful method in computer vision and pattern recognition because it determines the distance between each object point and the closest boundary. The binary image determines the distance between each pixel and the closest nonzero pixel in the distance transform. Euclidean norm is satisfied to use in this study which helps determine the straight-line distance between pixels to pixels and evaluated the measurement of specific points of the image. In the 2D Euclidean geometry, from the Cartesian coordinate, distance between 2 points with start point is *w*_*i*_ = (*w*_1_, *w*_2,_*w*_3,_ ⋯ *w*_*n*_) and the endpoint is *u*_*i*_ = ( *u*_1_, *u*_2,_*u*_3,_ ⋯ *u*_*n*_) following the Pythagorean theorem which is defined as

(2) $$\begin{array}{c} d\left({\text{w}}_{i},u_{i}\right)=\sqrt{\overset{n}{\underset{i=1}{\sum }}{\left(u_{i}-{\text{w}}_{i}\right)}^{2}}. \end{array}$$

The image provides the original dimension with *H* × *W* pixels, which are transferred as dimensional Euclid, namely, image space. Each pixel is represented as a point in the image space. Since the image space algebra can be conveniently expressed as seen above, the Euclidean distance of images can be calculated using metric coefficients *h*_*ij*_ which are defined as

(3) $$\begin{array}{c} h_{ij}=<g_{i},{\text{g}}_{j}>=\sqrt{<g_{i},{\text{g}}_{i}>}\sqrt{<g_{j},{\text{g}}_{j}>}*\cos\theta_{ij}, \end{array}$$

where <, > is the scalar value, and *θ*_*ij*_ is the angle between *g*_*i*_ and *g*_*j*_. All the pictures with checked landmarks and constructs were saved as noncompressed TIFF files. These all files were set to millimeters and analyzed with the same metric coefficient. In frontal view, the anthropometric ratios used to estimate intranasal symmetry [51, 52] were nasal height (the glabella to the subnasal) to width ratio, described as the distance between the maxilla-frontal right and left, ratio of mid-alar width shown as mid-alar-right to mid-alar-left, ratio of nasal base width shown as sub-alar-right to sub-alar-left, and total nose width from alare-right to alare-left, finally, the angle ratio between the dorsum's long axes and the midline ratio in alar asymmetry (Figure 1). The frontal process of the maxilla can also have flat, convex, or concave forms. In the lateral view (Figure 3), the research focused primarily on the tangent and angle that follows the nasal dorsum. Facial landmarks are collected automatically by the CNN model which helped to describe and predict of nasal bones based on these angular measurement. Measurement had been implemented by nine angles on facial skin and four angles on nasal bone. On facial skin, based on keypoint, every 3 identified keypoints in the lateral image could be defined as an angle. The nasofrontal angle, nasofacial angle, and nasomental angle shown in Figure 3(a) and other angles shown in Figure 3(b) described the morphology of the nose in general. The kyphion angle shown listed is the special angle that indicates the dorsal hump of nasal; it just appears in some specific participants.

### 3.2. Nasal Bone Properties

The nasal bones are two small bones which are supported by the bony septum body and are situated in the upper-middle of the vertical axis [52]. It is in charge of the shape of the nose or its corrective appearance, nasal bones has 4 borders: superior, medial, lateral, inferior namely, caudal edge of nasal bone known as rhinion, nasofrontal sature border which its top place called glabella, and lateral limited by nasomaxillary satures. Rhinion is where the nasal bones meet the cartilage; in different people, this bone will develop differently; it is considered a recognizable part of the hunchback of the bone and the cartilage layer slipped onto each other or mismatched. The keystone region shown in Figure 4(b) depicts the association of the bone irregularities and cartilaginous frameworks described by the kyphion. The kyphion angle listed in Table 2 is usually known as dorsal humps. These anomalies may result in a hump in the shape of a person's nose, rather than a flat slope from the bridge to the tip. A dorsal hump may also form as a result of trauma or accident. A bruised or fractured nose can cause a dorsal hump if the cartilage and bone heal unevenly. It is an essential anatomical structure that provides cohesion at the osseocartilaginous junction [9] and nasal bone analysis based on anthropometry is required to predict morphology of the nose through specific facial landmark.

The correlation between anthropometric indicators of the nasal bone has been analyzed and recorded from Vietnamese cadavers. The sizes of the nasal bone were measured by horizontal and vertical planes. In the horizontal plane, *d*3, *d*4, and *d5* shown in Figure 4(a) described the upper width of the nasal bone, the lower width of nasal bone, and the narrowest, respectively. On the other side, the narrowest segment of the nasal bone is considered when its location would above the eye and equal to or below the sellion (S). The average length of the nasal bone (N-R) is described by *d*2 in the vertical plane. There are the correlation between the upper widths with the narrowest segment of the nasal bone; the correlation between the distance from nasion (N) to sellion, the distance from sellion to rhinion (R), and the distance from S to Kyphion (K) at nasal hump when it possible seen. Last but not least, in the lateral view (Figure 4(b)), four angular dimensions included the nasion angle, dorsal profile angle, rhinion angle, and kyphion angle shown in Table 2 have been implemented for determining the nasal shape and also showing the relationship between the nose surface and the inner bony which separated by the thick of skin layer and the other factors.

One of the most important factors to consider when conducting rhinoplasty is skin thickness. The upper half of the nose's skin is thinner and flexible, while the lower half is thicker and more adherent. Analyzed from 33 adult cadavers, average skin thickness was noted to be greatest at the nasofrontal suture in which 1.25 ± 1.22 mm and least 0.6 ± 0.5 mm at the rhinion. Alharethy et al. [48] noted that the mean overlying skin thickness at the nasion was 3.89 ± 1.48 mm and at the rhinion was 1.16 ± 0.6 mm. The reason might be any nasal changes associated with ages and races (e.g., nasal lengthening or tip droop) can be caused by changes in the soft tissue that covers the nose.

## 4. Hybrid of Convolutional and Back-Propagation Neural Network

With the above preprocessing, augmentation, and partitioning of the nasal and facial anthropological datasets, the CNN and BPNN architecture especially for the morphological regression of the nasal bone is proposed. In this stage, CNN obtained the top results in many complicated classification and regression tasks. First of all, the original image was well prepared like described above. The augmentation and preprocessed images continually jointed the convolutional network as the input. The convolution network structure classifies facial keypoint into 29 points on the face in frontal, lateral, and basal images, which is shown in Figure 5. The labeled images on 3 perspective views were fed to each feature extractor to obtain the feature map separately. Various networks, such as ResNet, Inception, MobileNet, DenseNet-264, and VGG can be used as feature extractors, and feature maps of different dimensions can be obtained according to each network's structure. ResNet is a method consisting in adding feature maps, while DenseNet is a structure that concatenates feature maps. In this study, five models are used to extract features by continuously connecting the feature map of the previous layers with the input of the next layer in order to compare the efficient of extract feature map. Figure 5 shows CNN architecture in short nineteen layers with 16 convolution layers, 3 fully connected layers, 5 MaxPool layers with stride 1, and a Softmax layer. For all models, an Adam optimizer with learning rates 0.001 over 100 epochs is used. A batch size of 100 is used, with a validation split of 0.2. Each layer of the first convolution layer has a filter size of 3 × 3 for each layer. For each subsampling, the first pooling size of 3 × 3 and the next pooling size of 5 × 5 are replicated. After each max-pooling layer, a dropout is created. The dense layer is applied after the layer has been flattened.

The vanishing gradient can be improved, and feature propagation can be enhanced using this architecture. The depth of the feature map derived using all five networks is calculated by the growth rate and number of layers in each block, while the width and height are determined by the number of downsamplings. Since a pretrained network was used in this analysis, an input image of 224 × 224 × 3 is transformed into a feature map of 14 × 14 × 512 after filtering through the feature extractor. Each feature map from the 3 perspective images is converted into a vector using global average pooling and then concatenated into a single vector using concatenation. A dense layer is being used to perform the final classification. Pytorch was used to design the proposed network.

In this study the input image is set to *W* × *H* × *C* where *C* is number of channels and Width × Height (*W* × *H*) is the input dimension. The input image is given as an input to the first convolutional layer with filter (3 × 3) of size with rectified linear unit (ReLU) activation function. Output will be of the size (*W* − *H* + 1)  × (*W* − *H* + 1). It is essential to sum the contributions from the previous layer cells, weighted by the filter components, add a bias term, and then apply the activation function. The second convolutional layer was created using the same technique. The contribution of each convolutional layer was calculated using

(4) $$\begin{array}{c} F_{ab}^{k}=\sigma \left(\overset{m-1}{\underset{i=0}{\sum }}\overset{m-1}{\underset{j=0}{\sum }}\left({\text{w}}_{ij}x_{\left(a+i\right)\left(b+j\right)}^{k-1}\right)+\text{bias}\right), \end{array}$$

where *m* is a number of neurals in the *k* − 1 layer. The max-pooling layer takes a (*k* × *k*) region and outputs a single value which is the maximum for that region. The input layer is (*n* × *n*) layer, and the output will be a (*W*/*k*) × (*n*/*k*) layer, as each (*k* × *k*) block is reduced to just a single value via the max function.

(5) $$\begin{array}{c} \frac{\partial L}{\partial w_{ij}}=\overset{w-h}{\underset{a=0}{\sum }}\overset{w-h}{\underset{b=0}{\sum }}\frac{\partial L}{\partial x_{ab}^{k}}\frac{\partial x_{ab}^{k}}{\partial w_{ij}}, \end{array}$$

where *L* is a specified error function. The partial of *L* with respect to each neuron output is the error that needs to compute for the previous layer. The gradient component for each weight is given below function using the chain rule (6):

(6) $$\begin{array}{c} \frac{\partial L}{\partial x_{ab}^{k}}=\frac{\partial L}{\partial y_{ab}^{k}}\frac{\partial y_{ab}^{k}}{\partial x_{ab}^{k}}=\frac{\partial L}{\partial y_{ab}^{k}}\sigma^{\prime }\left(x_{ab}^{k}\right). \end{array}$$

Two convolutional layers have been configured to fully connect the dense layer and dropout layer of threshold 0.25. Since there are more than two output classes, the output layer has been used with the Softmax function. After initializing the Softmax at the output classes, the position of keypoints will be represented by a vector of two components, as seen in Figure 5. Keypoints are extracted from image as the feature map; each point would show by the position in 2D coordinate, represented by (*x*_*i*_, *y*_*i*_). Next stage, these points were used to calculate the distance in pair and angles as described in Section 3; for instance, alar base width would be calculated by the dimension between alar right (*x*_14_, *y*_14_) and alar left (*x*_16_, *y*_16_). The nasal width is correlated with the dimension between nasomaxillary sature at right (*x*_4_, *y*_4_) and nasomaxillary sature at left (*x*_7_, *y*_7_), etc. The distance method is implemented as the same on the cadaver's nasal bone dataset during surgery. After all, the nose distance of the participant and their morphology combined on nasal bone dimension of the cadaver with their nose morphology yet operation are continuing as the input of the special back-propagation which described in Figure 6.

First known, the internal organs in the human body will have a structure that self-regulates to suit the person's condition; the nose is no exception, since more tissue maintenance requires more oxygen consumption. The human nasal cavity may be connected to the slight mass of the body. For example, as compared to females, modern human men had a larger airway width and a larger lung capacity proportional to bodyweight (Hopkins and Harms, 2004). This is most likely related to well-established features of sexual dimorphism in regular energy and oxygen demands in Homo sapiens genders (Panter-Brick, 2002). Sexual dimorphism in these characteristics is most common throughout puberty, when adolescents begin to experience considerable increases in body mass, changes in body composition, and related changes in oxygen consumption needs (Bitar et al., 2000; Maynard et al., 2001; Wells, 2007). For these reason, BPNN has been used to predict the bony based on the prediction of all above factors. The BPNN is a fully connected neural network with 3 layers shown as Figure 6: an input layer, a hidden layer (or multilayers), and an output layer. This neural network will perform two main functions: forward and backward propagation. For modification of weight with optimized and precious reach at peak, each hidden layer would add a bias which allows update data training. The activation function named a rectified linear unit abbreviated by ReLU was added in the hidden layer attaches a weight to an input signal during forward propagation, after that the weighted signal is then forwarded to the output layer for calculation of the desire value. The ReLU function employed in this stage is described by (7) formula:

(7) $$\begin{array}{c} f\left(x\right)=\left\{\begin{array}{c} x\text{ if }x>0,\\ 0\text{ if }x\leq 0. \end{array}\right. \end{array}$$

The ReLU and its derivative also are monotonous. Whether it gets any negative input, it returns 0; however, when input receives any positive value *x*, it returns value. As a result, it produces an output with a value range of 0 to infinite. Successful completion of forward propagation or backward propagation would be allowed if the discrepancy (error) between the output value and the target output value reaches the tolerable error range. The biases and the weights in the BPNN are defined by output (8) function:

(8) $$\begin{array}{c} \text{BW}=f\left|\overset{n}{\underset{i=1,j=1}{\sum }}W_{ij}-{\text{bias}}_{ij}\right|, \end{array}$$

where *ij* is itinerary during training process. Learning rate is denoted by *f* and derivative of error with respect to weight was calculated by bias_*ij*_ = *∂*Error/*∂W*_*ij*_. Regarding recurrent training, the BPNN consistently changes the cost of the weight and bias vector, which gives the precise morphology of the nasal bone of the neural network close to the expected value shown in the target layer. By the result, the nasal bone can be classified into 5 classes which are represented in the result. The nasomaxillary sutures initially descended vertically and obliquely described as Type A. Type B, in which the nasomaxillary sutures were concave in the middle part. Type C, in which the frontonasal suture was relatively narrow and the nasomaxillary suture descended obliquely; Type D in which the frontonasal suture was relatively wide and the nasomaxillary sutures were concave in the middle part. Type E, in which the frontonasal suture was relatively wide and the nasomaxillary sutures descended vertically.

## 5. Results and Discussion

This section describes the training configurations and evaluation metrics used for performance analysis. The results of the architecture for facial masked segmentation, keypoint detection, and bone shape regression are discussed individually according to their sequence of the body index. The convolution proposed could predict facial keypoints with several deep learning models. Using predictive data from the CNN network as input data for the BPNN to modify the nasal bone morphology and performed by visual result in this section and evaluating the relationship between them most objectively.

### 5.1. Photogrammetric Evaluation and Performance Indicators

After labeling the entire dataset, the entire image and argumentation will be fed into the CNN to perform the learning of the parameters shown as Figure 7. Evaluating the model accuracy is an essential part of the process in creating machine learning models to describe how well the model is performing. The score function helps to measure regression performance listed as the mean absolute error (MAE), *R*-squared (*R*^2^), and mean average precision (mAP). The MAE is the average of the absolute difference between forecasted values and actual measured data, calculated by averaging the absolute difference over the selected dataset which is described by

(9) $$\begin{array}{c} \text{MAE}\left(y,\hat{y}\right)=\frac{1}{n}\overset{n-1}{\underset{i=0}{\sum }}\left|y_{i}-{\hat{y}}_{i}\right|, \end{array}$$

where ${\hat{y}}_{i}$ is the predicted value of the *i*^th^ keypoint and value of dimension, while *y*_*i*_ is corresponded the true value of keypoint location on face. *R*-squared is used to calculate the error between the predicted bounding boxes and the anchor boxes; improving localization loss will help detect objects become more accurate. The *R*^2^ represents the correlation between the predicted results and the actual output, varying from 0 to 1, as shown in equation (10):

(10) $$\begin{array}{c} R^{2}=1-\frac{{\text{SS}}_{\text{Regression}}}{{\text{SS}}_{\text{Total}}}=1-\frac{\sum_{i}{\left(y_{i}-{\overset{\wedge }{y}}_{i}\right)}^{2}}{\sum_{i}{\left(y_{i}-{\bar{y}}_{i}\right)}^{2}}. \end{array}$$

The closer the absolute value of *R* is to 1, the better the mode. A model with higher *R*^2^ values but lower MAE values performs better. In general, higher *R*^2^ values may coincide with smaller MAE values. Finally, mAP is usually used as the evaluation index of target detection performance. The mAP value is the region under the P-R curve, where recall is the *x*-axis and accuracy is the *y*-axis. mAP reflects the average accuracy of specific categories and can be used to evaluate the network model's performance in all categories. The mAP determination formula is as follows:

(11) $$\begin{array}{c} \text{mAP}=\frac{1}{k}\overset{k}{\underset{i=1}{\sum }}\int_{0}^{1}\text{PdR}, \end{array}$$

where *k* represents number of detected categories. *p*_*i*_ and $\overset{⌢}{p_{i}}$ are detected keypoints by algorithm of deep learning and manual measurement method, respectively.

### 5.2. Training Configuration and Keypoint Detected Results

A green fabric background was used to easily facial segmentation making it possible for the pixels to receive only in the face of the object according to different angles and reduce variance in computation complexity. Normalize and augment data had been shuffled to detect and localize all essential landmarks. Several state-of-the-art detectors that are based on convolutional neural networks have been tested and validated performed in Figure 8. Following the output of a number of CNN layers for facial segmentation, the keypoint filters are performed as part of the data normalization procedure to better align the images in an upright pose. Similar to facial segmentation, applied multiple state-of-the-art model for facial keypoint detection were compared best model to any optimally rotating nasal anthropology photographs. Training and testing the detection of nasion point (deepest and hardest point) on the face were illustrated with various network models to meet the requirements in rapid and precise training. MobileNet with dropout was configured with a total of 4,253,864 parameters. The learning rate was 0.001 for training this model; the loss for MobileNet with the dropout layer indicates a significant reduction in loss performed. Figure illustrates how a learning rate of 0.001 reduces failure across epochs. It can be seen in Table 3 and Figure 8 that the DenseNet model has returned smaller MAE than InceptionV3 and ConvNet, which were 1.738 mm and 3.412 mm, respectively. It because the original implementation only utilizes two-layer skip connection and without any shuffle or deeper channel learning. Therefore, ConvNet with dropout predicts key-points less accuracy than DenseNet and InceptionV3, and the worst for applying in this study. VGG19 model has the loss value slowly converged to desire value at first one fourth of 100 epochs, after that it was stable and reached the optimal value, however, it could meet by overfitting when the training process continues at the same with other.

As a result, when comparing to a basic skip connection scheme, the three layers of the residual module with a larger kernel in the middle layer provides better keypoint detection. Some predicted keypoints on the face are missing and do not perform well with the head orientation, which is helpful if the head angle is approximate. It is worth nothing that depthwise and pointwise convolution in the MobileNet has produced excellent task of detection all keypoints even though the model parameter of was used as the lighter than another. By the way, rather than just the later layers, the early layers will play an important role in learning the best feature representation. Therefore, according to overall result performance, MobileNet is selected as the best model for landmark detection due to its low MAE values and lightweight (less than 4 million parameters).  Figure 9 was shown samples of detection of keypoints with belong accuracy belong accuracy in three directions that fed to nasal bony regression network. From Table 4, the model applied MobileNet has shown quite good results for average loss at 0.1199% with 29 complex landmarks. The mAP accuracy in the testing of dataset for pictures of automatic cameras, or images with simple backgrounds with full light, is quite high 97.869%. However, the input image is heavily affected by the surroundings and lighting, the model accuracy drops sharply to 85.739% while model have being trained with the original and augment images.

### 5.3. Evaluate Nasal Morphology Based on Anthropology and CNN-BPNN

In this research, analysis on 33 cadavers was used to examine the nasal bone morphology. Females made up 45.5% of the dataset, with an average of 65. With the nasal bone having *K* point ratio accounted for 24.2%. The sample with *K* points are found in the middle of the dorsal was 75%. Vietnamese nasal bone length calculated by the distance start from N to R, which average value was 23.81 ± 2.94 mm, while the average distance between nasion and the deepest point of nasal bone was 5.71 ± 1.22 mm. Finally, distance from sellion to rhinion was 18.56 ± 2.69 mm.

At the nasion, the bone width between two left and right borders are 5.52 ± 1.34 mm and 5.59 ± 1.31 mm, respectively. Similarly, linear distances have been measured (shown as Table 5) at the lowest point—sellion (S) in the dorsal line and rhinion (R). Bone's width at the S is the smallest distance which is 5.05 ± 0.84 mm at the left and 5.17 ± 0.95 mm at the right. The average length of the nasal bone (N-R) is 23.81 ± 2.94 mm. The nasal bone width on average is 10.21 ± 2.53 mm; the lower nasal bone width is 17.08 ± 2.08 mm. The narrowest piece of the average horizontal nasal bone is 8.24 ± 1.58 mm. However, there are no variations in bony sizes based on gender or age, despite the fact that nasal anthropology would change in distance or angle by using CNN to detect and measure. By this exam, nasal bone morphologies are divided into two categories: direct front view and lateral view. At first, Lang and Baumeister [38] categorized German bone shape into eight groups in frontal view. However, category was too complicated, Hwang et al. [39] has shortened categories into 5 types when studying Korean nasal bone shape, and this shortened classification was being widely applied in numerous studies. Based on the distance calculated above, result of the nasal bone morphology of our study was shown in Table 6. The category illustrated that most of nasal bones of Vietnamese with direct perspective. Type A was present in 57.6% of participants. Type B was present in 30.3% of the noses. In particularly, types C, D, and E were not common form; the remaining types account for a very low proportion. By this category, nasal shape following each race would have differed characteristics which was performed in Table 7. For instance, types D and E were not observed in Koreans. These results were different from the study carried out in Germans, in which type A was most common (68.3%), while types B, D, and E comprised the rest at an equal frequency of 10.1% in each case.

In the lateral view, the shape of the nasal bone had classified follows its angle measurement by Sugawara. His result showed the majority of nasal bone ratio was “S” type with 88% in Caucasian race [42]. The big different of V-shaped nasal bones and S-shaped nasal bones was the curve line that nasal structure make from. “V” type nasal morphology has a straight line structure across sellion through rhino and consequently single point of angulation at the dorsal profile angle (DPA), while “S” type nasal morphology has a curving arc that starts at sellion, travels through a distinct point at kyphion, and peaks at rhino. There are two angulation locations, one at the DPA and one at the kyphion angle. Meanwhile, the majority of Vietnamese nasal bone shape had “V” shape (78.8%). The reason caused of nasal shape was depended on the hump analysis shown in Table 8. Besides, it can be seen that the majority of Europeans are “S” shape, while Vietnamese had the other. This may stem from racial differences leading to completely different nasal bone structure characteristics. The size and the shape of the nasal bone can be used to clarify the anthropological characteristics of each race.

The second experiment the work of BPNN is implemented on 182 participants, from an average age of 22.01 ± 1.39, with 55.5% female. Predicted data is also used to visualize nose shape that appropriate with the predicted nasal bone dimension. The experimental results of BPNN combined with topology are shown in Figure 10. The detected data is described as a frequency and percentage with qualitative variables. Medium and standard deviation was described with quantitative variables. Since the index of each individual is different, statistical analysis is applied to test the result correlative between nasal bony and the other nose's dimension. *T*-test analysis was used to determine gender differences and the difference in nutritional status in indicators such as BMI, Kruskal-Wallis test replaced *T*-test in some results. In participant's data, the overweight and obesity rate was quite high at 19.2% and 20.3%, respectively. The rate of normal weight still accounted for 52.8%. Most sizes of nasal root areas of the study sample have the difference between men and women, in which the measurements in men are larger than women. Accordingly, the study shows that people with high BMI will have shorter than in height of the nasal but the nasal width is wider than low BMI shown in Table 9. All soft tissue angles were significantly larger than the bone angles for the nasofrontal angle, nasal tip angle, and nasolabial angle, respectively. With regard to sex, the bone and soft tissue nasofrontal angles were significantly larger in women than in men, whereas the bone and soft tissue nasal tip angles were significantly larger in men than in women. The nasolabial angle showed no significant difference between men and women (bone, *p* = 0.002; soft tissue, *p* = 0.005).

When comparing the size of nasal radix according BMI, there is a statistically significant difference following Table 8. Dorsal length (n–prn) was greater in underweight and normal weight groups than the overweight-obese (*p* = 0.047). Nose base width (al–al) and nose swing width (ac–ac) of the underweight and the normal weight would be narrower than the others by *p* = 0.001 and 0.024, respectively. The distance between nasion and rhinion (n–r) would be greater in slim and normal people than in overweight–obesity (*p* < 0.001). Subnasale and pronasale distance (sn–prn) would be smaller in the underweight and normal groups than in the overweight-obese group (*p* = 0.02).

Table 10 depicted the difference in sexual dimorphism, and nasofrontal angle average was 136.410 ± 7.990, with females having a greater angle than males. The middle face (distance from nasion to subnasale) accounts for roughly 43% compared to the length of the face from the nasal radix to the chin at the lowest point (n-gn) and has a gender difference, with the female having a greater rate than the male.

## 6. Conclusions

In this paper, for medical image analysis, we proposed a hybrid of CNN and BPNN on detecting facial landmarks and predict nasal morphologies with 2D digital image. We have shown that the power the proposed architecture can be harnessed to provide fast and accurate solutions to automatically identify anthropology keypoints and specific nasal distance. The comparison of the proposed CNN with optimized state-of-the-art approaches evaluated with five distinct attack architecture models demonstrated MobileNet predominance under many circumstances. According to anthropological studies, nasal morphology is influenced by various factors could be known as BMI, age, gender, and race. These features are being selected as a part of the input layer of our back-propagation neural network which increases the predicted efficacy. Moreover, based on the latest studies of nasal morphology, Vietnamese nasal morphology could be divided into various types in different perspective views known as frontal view and lateral view.

This study not only focuses on the application of CNN and BPNN identifies facial anthropology on nasal bone shape regression but also show a number of clinical analysis and applications. Aesthetic surgeons when planning surgery needs to discriminate indicators features of the patient's nose on the soft tissue which has relevant relationship to the bone. Otherwise, the correlation between these indicators helps the surgeon when intervening should pay attention to the harmony between the structures of the nasal bone. Combined altogether, the current study provides knowledge on the nasal anthropology and morphological features in the Vietnamese population, which could be used to identify the Vietnamese anthropological traits.

## Figures and Tables

**Figure 1:** Anthropometric landmarks have been indirectly measured in three perspective views; all dimensions are in millimeters (mm) based on split length on the ruler belongs with an image. Image modified with permission. tr: trichion; g: glabella, s: sellion; r: rhinion; en: endocanthion; ex: exocanthion; mf: maxillofrontale; prm: pronasale; al: alare; ac: subalare; sn: subnasale; zy: zygion; li: labrale inferius; ls: labrale superius; ch: cheilion; pg: pogonion; gn: gnathion.

**Figure 2:** The framework of proposals in nasal bone shape prediction.

**Figure 3:** Angular measurements based on indirect anthropology on the patient's skin with angular measurement to be listed as (a) g-n-prn, n-prn-pg, g-sn-pg, n-prn-sn and (b) n-prn-sn, cm-sn-ls, li-sm-pg, g-sn-pg. Image used with permission of subject.

**Figure 4:** Distances are practically measured for the nasal bones, in which horizontal *d*4, *d*5, and *d*3 are the width of nasal bones at the nasomaxillary suture line, nasion, and nasofrontal suture, perspectively. With red line, it illustrated the distance between nason and sellion (dimensions are shown in mm) (a). Nasal bone had been removed, ligament and soft tissue captured from the right side (b).

**Figure 5:** Proposed convolutional neural network (CNN) model for anthropological localization.

**Figure 6:** Proposed BPNN model for nasal bone morphology prediction.

**Figure 7:** Features extracted in output layer and representation of feature map in every CNN's layer.

**Figure 8:** Accuracy and lost performed of detecting keypoint by 5 different network models over a certain period.

**Figure 9:** Anthropometric keypoints have been predicted by CNNs model in three perspective views; (a, c) frontal, lateral, and basal views, respectively. All dimension units are in millimeter (mm) based on split length on the ruler belongs with an image can be automatically measured.

**Figure 10:** Nasal morphology was presented in the lateral image with back-propagation, including the bounding on nose shape and approximately size of nasal bone.

**Table 1:** Characteristics and standard parameter for input training and validation by 3 specific groups.

Characteristic	Training group	External evaluation group	Internal evaluation group
	(*n* = 2000)	(*n* = 182)	(*n* = 33)
Male	88	81	18
Female	1912	101	15
Age	35.09 ± 11.56	22.01 ± 1.39	64.9 ± 13.9
BMI	24.86 ± 10.43	22.34 ± 12.8	N/A

Mean ± standard deviation. N/A: not available.

**Table 2:** The nasal angles on the skin surface are listed from 1 to 9 and the measurement angles are made on the nasal bone from 10 to 13.

No.	Abbreviation	Name
1	g-n-prn	Nasofrontal angle
2	pg-n-prn	Nasofacial angle
3	g-sn-pg	Facial angle
4	n-prm-sn	Nasomental angle
5	n-prm-cm	Nasal angle
6	cm-sn-ls	Nasolabial angle
7	*α*	Middle facial height angle
8	*β*	Lower facial height angle
9	n–k–r1	Nasal kyphion rhino
10	NA	Nasion angle
11	DPA	Dorsal profile angle
12	KA	Kyphion angle
13	RA	Rhinion angle

^1^k: kyphion. This feature appeared in some cases, affecting the shape and profile of the nose.

**Table 3:** Performance of CNN-BPNN predicting facial landmarks and its morphology applied from five CNN models.

Evaluate metrics		ConvNet	InceptionV3	MobileNet	DenseNet	VGG19
Training and validation stage	*R* ^2^	0.582	0.836	0.957	0.884	0.919
	MAE (mm)	2.323	1.529	0.176	0.631	0.352
Testing stage	*R* ^2^	0.331	0.749	0.934	0.912	0.871
	MAE (mm)	3.412	1.738	0.281	0.442	0.597

**Table 4:** Algorithm accuracy in the best model construction process.

	Training	Validation	Testing
mAP	98.2258%	98.5326%	97.8693%

**Table 5:** Nasal bone distances indirectly measured comparing with custom measured values following sexual dimorphism.

Predicted nasal distances	Male (*n* = 81)	Female (*n* = 101)	Average value	*p* mean
N–S	5.56 ± 1.25	5.89 ± 1.19	5.71 ± 1.22	0.452
S–K (*n* = 8)	14.54 ± 0.73	14.08 ± 0.93	14.31 ± 0.82	0.461
K–R (*n* = 8)	4.61 ± 1.29	4.52 ± 1.08	4.56 ± 1.10	0.917
S–R	18.85 ± 3.02	18.22 ± 2.29	18.56 ± 2.69	0.515
N–R	23.79 ± 3.46	23.83 ± 2.29	23.81 ± 2.94	0.971

Each value is represented as mean ± standard deviation in millimeters;.

**Table 6:** Nasal bone morphological regression and classification by the frontal view in our study.

Nasal morphology	Male (*n* = 18)	Female (*n* = 15)	Percentage
Type A	9 (50.0)	10 (66.7)	57.6%
Type B	6 (33.2)	4 (26.7)	30.3%
Type C	1 (5.6)	0	3.0%
Type D	1 (5.6)	1 (6.6)	6.1%
Type E	1 (5.6)	0	3.0%

**Table 7:** Comparison of the present nasal bone data with the previous studies carried out in other races.

Author	Race	A (%)	B (%)	C (%)	D (%)	E (%)
Present study	Vietnamese (33)	57.6	30.3	3.0	6.1	3.0
Lang and Baumeister [38]	German (79)	68.3	10.1	1.3	10.1	10.1
Hwang et al. [39]	Korean (88)	43.2	52.3	4.5	0.0	0.0
Prado et al. [53]	Brazil (97)	49.5	27.8	13.4	2.1	7.2

**Table 8:** Nasal bone shape from angular regression values in the lateral view (*n* = 33).

	“V” shape (*n* = 26)	“S” shape (*n* = 7)
Male	15 (83.3)	3 (16.7)
Female	12 (80.0)	3 (20.0)
With the kyphion	1 (12.5)	7 (87.5)
Without the kyphion	25 (100)	0 (0)

**Table 9:** Nasal dimension are predicted following body mass index (BMI).

No.	Predicted nasal distances	Underweight	Normal weight	Overweight	Obesity	*p* mean
		≤18.5	(18.5-24.9)	(25-29.9)	(over 30)	
1	n–prn	4.03 ± 0.33	3.85 ± 0.37	3.92 ± 0.49	3.73 ± 0.34	0.047
2	n–sn	4.90 ± 0.34	4.91 ± 0.31	4.96 ± 0.33	4.88 ± 0.47	0.496^∗^
3	al–al	3.90 ± 0.29	4.01 ± 0.31	4.19 ± 0.38	4.19 ± 0.27	0.001
4	ac–ac	3.14 ± 0.33	3.23 ± 0.29	3.33 ± 0.37	3.38 ± 0.29	0.024
5	n–r	1.36 ± 0.22	1.26 ± 0.21	1.24 ± 0.20	1.12 ± 0.19	0.0006
6	en–en	3.60 ± 0.27	3.57 ± 0.23	3.68 ± 0.26	3.68 ± 0.25	0.052
7	sn–prn	1.50 ± 0.22	1.67 ± 0.19	1.70 ± 0.18	1.67 ± 0.18	0.020

^∗^Kruskal-Wallis method, Mean ± standard deviation.

**Table 10:** Nasal dimension are predicted based on sexual dimorphism.

No.	Predicted nasal angles	Male (*n* = 81)	Female (*n* = 101)	Average value	*P* mean
1	g–n–prn	133.89 ± 1.06	138.43 ± 0.57	136.41 ± 7.99	0.0003
2	n–prn–sn	103.43 ± 0.64	104.91 ± 0.60	104.25 ± 5.95	0.095

Mean ± standard deviation.

## Data Availability

These data are supporting of Pham Ngoc Thach University of Medicine. All data captured face of patients which is permitted to analysis but not including publish due to personal priority.
